# Resveratrol increases nucleus pulposus matrix synthesis through activating the PI3K/Akt signaling pathway under mechanical compression in a disc organ culture

**DOI:** 10.1042/BSR20171319

**Published:** 2017-11-23

**Authors:** Xiaorui Han, Xiaoming Leng, Man Zhao, Mei Wu, Amei Chen, Guoju Hong, Ping Sun

**Affiliations:** 1 Guangzhou First People’s Hospital, the Second Affiliated Hospital of South China University of Technology, Guangzhou, China; 2 Universal Medical Imaging Diagnostic Center, Guangzhou, China; 3 Department of Radiography, The First Affiliated Hospital of Clinical Medicine of Guangdong Pharmaceutical University, Guangzhou, China; 4 Guangzhou University of Chinese Medicine, and Biomedical Science School, University of Western Australia, Australia; 5 Department of Orthopedic, The First Affiliated Hospital of Guangdong Pharmaceutical University, Guangzhou, ChinInsert Affiliation Text Here

**Keywords:** matrix, mechanical compression, nucleus pulposus, resveratrol

## Abstract

Disc nucleus pulposus (NP) matrix homeostasis is important for normal disc function. Mechanical overloading seriously decreases matrix synthesis and increases matrix degradation. The present study aims to investigate the effects of resveratrol on disc NP matrix homeostasis under a relatively high-magnitude mechanical compression and the potential mechanism underlying this process. Porcine discs were perfusion-cultured and subjected to a relatively high-magnitude mechanical compression (1.3 MPa at a frequency of 1.0 Hz for 2 h once per day) for 7 days in a mechanically active bioreactor. The non-compressed discs were used as controls. Resveratrol was added along with culture medium to observe the effects of resveratrol on NP matrix synthesis under mechanical load respectively. NP matrix synthesis was evaluated by histology, biochemical content (glycosaminoglycan (GAG) and hydroxyproline (HYP)), and expression of matrix macromolecules (aggrecan and collagen II). Results showed that this high-magnitude mechanical compression significantly decreased NP matrix content, indicated by the decreased staining intensity of Alcian Blue and biochemical content (GAG and HYP), and the down-regulated expression of NP matrix macromolecules (aggrecan and collagen II). Further analysis indicated that resveratrol partly stimulated NP matrix synthesis and increased activity of the PI3K/Akt pathway in a dose-dependent manner under mechanical compression. Together, resveratrol is beneficial for disc NP matrix synthesis under mechanical overloading, and the activation of the PI3K/Akt pathway may participate in this regulatory process. Resveratrol may be promising to regenerate mechanical overloading-induced disc degeneration.

## Introduction

Patients with intervertebral disc degeneration (IDD) are commonly seen in the orthopedic clinic [1,2]. Previous studies has established that IDD largely contributes to individual disability due to the accompanying low back and leg pain [3]. Currently, the clinical treatment mainly aims to eliminate or alleviate symptoms but not to its pathogenesis. Despite the existing breakthroughs in the disc degeneration-related research, more basic researches are necessary to biologically regenerate the degenerative disc.

The intervertebral disc (IVD) locates between two vertebral bones and functions as a loading absorber and transmitter [4]. The IVD consists of three structurally integrated parts: the peripheral annulus fibrosus (AF), the central nucleus pulpous (NP), and the cartilage endplate (CEP) [5]. The normal mechanical function of the IVD mainly depends on the content and composition of disc NP matrix (proteoglycan and collagen II), which will be decreased and denatured during disc degeneration [6,7]. Therefore, maintenance of the normal NP matrix homeostasis is implicated for keeping the normal mechanical IVD function.

As a common external pathological factor of disc degeneration, mechanical compression affects NP cell from cellular fate to cellular biosynthesis [8]. Increasing researches have demonstrated that mechanical load plays an important role in disc development and degeneration [9]. Moreover, a physiological loading is necessary to keep active disc matrix self-renewal, whereas an unphysiological loading sharply destroys the balance of matrix metabolism and homeostasis [10,11]. Therefore, promotion of the disc NP matrix biosynthesis may be effective for retarding damaged disc function that was caused by mechanical overloading.

Resveratrol, a natural phytoalexin found in plants including peanuts and grapes, is reported to have a wide protective effects in different cell types, such as the anti-inflammatory, anti-aging, and cartilage protection [12]. Recently, two studies showed that resveratrol can stimulate the matrix metabolism (i.e. up-regulating mRNA of collagen II and aggrecan, and down-regulating mRNA of matrix degrading enzymes, such as MMP-3, MMP-13, and ADAMTS-4) [13,14]. In the present study, we mainly aimed to investigate the effects of resveratrol on disc NP matrix synthesis under a high-magnitude mechanical compression and the potential signaling transduction pathway in this regulatory process.

## Materials and methods

### Ethical statement

All experiments were approved by the Ethics Committee at Guangzhou First People’s Hospital [SDRY (GU) 2010-0045].

### Disc isolation and bioreactor culture

The intact discs from 13 healthy pigs (male, 10–12 kg, 3–4 months old) were isolated according the previous method [11,15]. Briefly, after animal killing via intravenous injection of an overdose of intravenous (100 mg/kg), the spinal column was separated and then the intact discs with CEP (Th11/Th12-L4/L5) were isolated under sterile conditions using a dissecting microscope. After all discs were rinsed with phosphate buffer solution (PBS), they were perfusion-cultured and compressed at a magnitude of 1.3 MPa (1.0 Hz, 2 h once per day) for 7 days in the mechanically active bioreactor that was described in a previous study [16]. The 1.3 MPa of compressive magnitude was designed as a high-magnitude mechanical compression because it has been demonstrated to significantly inhibit NP matrix anabolism and promoting NP matrix catabolism in a previous study [11]. Meanwhile, resveratrol (50 and 100 μM) [13,14] was added along with the culture medium to investigate the effects of resveratrol on NP matrix synthesis and PI3K/Akt pathway under this high-magnitude mechanical compression. The control discs were not compressed. A total of 100 ml of fresh DMEM culture medium (Gibco, U.S.A.) supplemented with 10% (v/v) fetal bovine serum (FBS, Gibco, U.S.A.), 1% (v/v) penicillin–streptomycin (Gibco, U.S.A.), 0.025 mg/ml ascorbic acid (Sigma, U.S.A.), and 15 mM HEPES (Sigma, U.S.A.) were circulated at a rate of 5 ml/min according to our own experience. Additionally, discs from the same levels were used for the same experiment to avoid the interference caused by different vertebral levels [17]. For example, the Alcian Blue staining assay was performed on the same three discs (Th11/12, Th12/L1, and L1/2) from different animals.

### Alcian Blue staining assay

Briefly, the cultured discs were rinsed with PBS. Then, they were fixed with 4% paraformaldehyde, decalcified with 10% ethylenediaminetetraacetic acid (EDTA), and embedded in paraffin. After 5 μm thick cross-sections were prepared, Alcian Blue assay was performed. All sections were observed under a light microscope and the staining intensity was quantified using Image-Pro Plus software (Version 5.1, Media Cybernetics, Inc.).

### RNA extraction and real-time PCR analysis

Gene expression of SOX-9 and NP matrix macromolecules (aggrecan and collagen II) was analyzed in the present study. Briefly, after the total RNA was extracted from the isolated NP tissue using the Trizol Reagent (Invitrogen, U.S.A.) and synthesized into cDNA using PrimeScript™ II 1st Strand cDNA Synthesis Kit (TaKaRa, Japan). Then, the PCR reaction was perform on a reaction mixture (20 μl) containing 10 μl of SYBR Green Mix (TOYOBO, Japan), 7.5 μl of RNase-free water, 1.5 μl of cDNA, and 1μl of primer mix. The thermal cycling for all reactions was as follows: 5 min at 95°C, followed by 35 amplification cycles of 30 s at 95°C, 20 s at 56°C, and 15 s at 72°C. Gene specific primers (Table 1) were designed and synthesized by a domestic commercial company (Sangon, Biotech Co., Ltd., China). GAPDH was used as an internal control. The method of 2^−ΔΔ*C*^_t_ was used to calculate the relative gene expression of target genes.

**Table 1:** Primers of target genes

Gene	Accession number	Forward (5′–3′)	Reverse (5′–3′)
GAPDH	NM_001206359.1	ACCTCCACTACATGGTCTACA	ATGACAAGCTTCCCGTTCTC
SOX9	NM_213843.1	TGCTGAATGAGAGCGAGAAG	CGCGGCTGGTACTTGTAAT
Aggrecan	NM_001164652.1	CGTGGTCCAGCACTTCTAAA	AGTCCACTGAGATCCTCTACAC
Collagen II	XM_001925959.4	CCGGGTGAACGTGGAGAGACTG	CGCCCCCACAGTGCCCTC

### Immunohistochemical staining assay

Immunohistochemistry was performed on the disc tissue slices to investigate matrix protein (aggrecan and collagen II) deposition. Briefly, after the sections undergo dewaxing, inactivation of peroxidase, antigen retrieval with stomach protease, and blockage with 5% FBS, they were incubated with primary antibodies against aggrecan (Norvus, NB120-11570, diluted 1:200) and collagen II (Abcam, ab34712, diluted 1:200) at 4°C overnight, followed by the incubation with corresponding HRP-conjugated secondary antibodies (goat anti-mouse IgG and goat anti-rabbit IgG, ZSGB-BIO, China, diluted 1:200). Then, all sections were incubated with the diaminobenzidine (DAB) to develop the positive staining. Finally, sections were observed under a light microscope (Olympus EX51, Japan) and the staining intensity was quantified using Image-Pro Plus software (Version 5.1, Media Cybernetics, Inc.).

### Western blotting assay

After culture, the discs were rinsed with PBS and the innermost NP tissue was isolated under a dissecting microscope. Then, Western blotting assay for SOX-9, aggrecan, and collagen II was performed. Briefly, after the total protein was extracted using RIPA lysis buffer (Beyotime, China), equal protein sample in each group was subjected to SDS/PAGE system and transferred to the PVDF membrane. Then, incubation of the primary antibodies (GAPDH: Abcam, ab8245; collagen II: Abcam, ab34712; aggrecan: Santa Cruz, sc-16492; SOX9: Santa Cruz, sc-20095; all were diluted 1:1000) was performed at 4°C overnight, and incubation of the corresponding HRP-conjugated secondary antibodies (goat anti-mouse IgG, goat anti-rabbit IgG, and mouse anti-goat IgG, ZSGB-BIO, China, diluted 1:1000) was performed at room temperature for 2 h. Thereafter, protein bands on the PVDF membrane were visualized using ECL Plus reagent (Thermo, U.S.A.). Then, protein expression normalized to GAPDH was calculated according to the gray value that was measured using the ImageJ software (National Institutes of Health, U.S.A.).

### Biochemical content measurement

NP tissue was isolated as described above and was used to measure glycosaminoglycan (GAG) and hydroxyproline (HYP) content. Briefly, one group of NP samples was lyophilized for 24 h and weighed to determine the dry weight. Then, the dried NP samples were digested at 60°C for 24 h in 1 ml of water containing 5 mg/ml papain, 0.2 mol/l NaCl, 0.01 mol/l cysteine hydrochloride, 0.1 mol/l CH_3_COONa, and 0.05 mol/L Na_2_-EDTA (Sangon, Biotech Co., Ltd., China). Then, the GAG content was calculated using a dimethylmethylene blue (DMMB) assay [18] in which chondroitin sulfate from shark cartilage was used as a standard. Another group of NP samples was weighed to determine their wet weights, and then the HYP content was determined using a HYP quantification kit (NanJing JianCheng, China) according to the manufacturer’s instructions.

### Statistical analysis

All data were expressed as the mean ± standard error of mean (SED). Each experiment was performed in triplicate to ensure repeatability. After the homogeneity test for variance, intergroup difference was analyzed by the one-way analysis of variance (ANOVA) using SPSS 17.0 software. The *post hoc* test was performed using the LSD test. A statistically difference was considered when the *P*-value < 0.05.

## Results

### Alcian Blue staining

The staining intensity of Alcian Blue is able to reflect proteoglycan content and distribution within the NP tissue [19]. Results showed that staining intensity in this high-magnitude mechanical compression group is significantly lower than the control group, whereas the addition of resveratrol partly increased staining intensity under the mechanical compression in a dose-dependent manner (Figure 1).

**Figure 1:** Histological observation. Alcian Blue staining of nucleus pulposus (NP) tissue; magnification = 200×, scale = 100 μM, *n*=3. Data are expressed as mean ± SD. *: significant difference (*P*<0.05) between two groups. #: significant difference (*P*<0.05) compared with the 1.3 MPa group.

### Gene expression

Aggrecan and collagen II are the main macromolecules of NP matrix and are transcriptional-regulated by the transcription factor SOX-9 [20]. Therefore, expression of all those three genes is important for NP matrix anabolism. Results showed that gene expression of these molecules was significantly down-regulated in this high-magnitude mechanical compression group compared with the control group, whereas the addition of resveratrol could obviously increase their expression levels (Figure 2).

**Figure 2:** Gene expression analysis. Real-time PCR analysis of nucleus pulposus (NP) matrix biosynthesis-related molecules (SOX-9, aggrecan, and collagen II). Data are expressed as mean ± SD. *: significant difference (*P*<0.05) between two groups. #: significant difference (*P*<0.05) compared with the 1.3 MPa group.

### Immunohistochemical staining

Immunostaining for aggrecan and collagen II showed that this high-magnitude compression significantly decreased their staining intensity compared with the control group. Addition of resveratrol was able to increase their staining intensity in a dose-dependent manner under the mechanical compression (Figure 3).

**Figure 3:** Immunohistochemical observation. Immunohistochemical staining of nucleus pulposus (NP) matrix macromolecules (aggrecan and collagen II) and its quantification; magnification = 200×, scale = 100 μM, *n*=3. Data are expressed as mean ± SD. *: significant difference (*P*<0.05) between two groups. #: significant difference (*P*<0.05) compared with the 1.3 MPa group.

### Western blot analysis

Western blot analysis of the activity of the PI3K/Akt pathway showed that activation of the PI3K/Akt pathway was significantly inhibited by this high-magnitude mechanical compression. However, addition of the resveratrol obviously increased its activity under mechanical compression in a dose-dependent manner (Figure 4A). Western blot analysis of NP matrix anabolism-related molecules showed that protein expression of the transcription factor SOX-9 significantly decreased in this high-magnitude mechanical compression group compared with the control group, whereas resveratrol partly increased SOX-9 protein expression in a dose-dependent manner under the mechanical compression. In addition, protein expression of aggrecan and collagen II showed a similar trend to that of SOX-9 (Figure 4B).

**Figure 4:** PI3K/Akt pathway activity and protein expression of matrix anabolism-related molecules. Western blot analysis of the activity of the PI3K/Akt pathway (**A**) and protein expression of nucleus pulposus (NP) matrix biosynthesis-related molecules (SOX-9, aggrecan, and collagen II) (**B**); magnification = 200×, scale = 100 μM, *n*=3. Data are expressed as mean ± SD. *: significant difference (*P*<0.05) between two groups. #: significant difference (*P*<0.05) compared with the 1.3 MPa group.

### Biochemical content

Both the GAG content and HYP content were significantly decreased under this high-magnitude mechanical compression compared with the control group. Addition of the resveratrol obviously increased their content in a dose-dependent manner under the mechanical compression (Figure 5).

**Figure 5:** Biochemical content measurement. Measurement of biochemical content within the nucleus pulposus (NP) tissue. (**A**) Glycosaminoglycans (GAG) content analysis and (**B**) hydroxyproline (HYP) content analysis. Data are expressed as mean ± SD. *: significant difference (*P*<0.05) between two groups. #: significant difference (*P*<0.05) compared with the 1.3 MPa group.

## Discussion

The stable matrix homeostasis with the disc NP tissue is important for the maintenance of normal disc mechanical function [21]. Matrix content decrease and matrix denaturation are two classical pathological features during disc degeneration [22]. As an initiating and inducing factor of disc degeneration, mechanical overloading is demonstrated to have a destructive effect on matrix anabolism while a stimulative effect on matrix degradation [8,10]. Hence, retaining the matrix synthesis is important for normal disc function under mechanical overloading. In the present study, we confirmed that mechanical overloading significantly inhibited NP matrix synthesis and demonstrated that resveratrol partly promoted NP matrix biosynthesis through activating the PI3K/Akt pathway under a high-magnitude mechanical compression. The present study provides potential therapeutic effects of resveratrol on mechanical overloading-induced disc degeneration.

Disc organ culture system is a suitable platform for studying disc biology due to its maintenance of the structural integrity and accurate controllability over the external physical and chemical factors [23]. Moreover, it is advantageous that the application of the perfusion bioreactor can make the present study more closer to the *in vivo* situations [24]. Previously, this perfusion bioreactor has been also described and used to culture tissue-engineered bone, cartilage, and vessel [16,20]. The magnitude of 1.3 MPa was designed as a high-magnitude mechanical compression because it can do harms to disc cell biology, such as promoting NP cell apoptosis and inhibiting NP matrix biosynthesis [11].

During disc degeneration, NP matrix proteins including proteoglycan and collagen II significantly declined, leading to the impaired disc mechanical function [22]. In the present study, NP matrix biosynthesis was obviously suppressed by this high-magnitude compression, reflected by the attenuated Alcian Blue staining intensity, down-regulated gene and protein expression of SOX-9, aggrecan and collagen II, and the decreased biochemical content (GAG and HYP). This is in line with previous opinions that mechanical overloading inhibits disc matrix synthesis and promotes matrix degradation [10], indicating that mechanical overloading is a risk factor of disc degeneration. Recently, many studies have investigated the potential mechanisms behind the mechanical overloading-induced attenuation of disc matrix biosynthesis, such as cell apoptosis, cell senescence, cell autophagy, and up-regulation of matrix degrading enzymes (MMPs and ADAMTs) [25–28]. However, the accurate molecular mechanisms need to be further studied.

Resveratrol is a natural phytoalexin found in various plants. Its effects of anti-inflammatory, antioxidant, and cardioprotective have been widely reported [12]. More recently, several studies have shown that resveratrol provides a protective effect on articular cartilage in rabbit models of osteoarthritis and rheumatoid arthritis [29,30]. Importantly, a previous study demonstrated that resveratrol injection significantly decreased loss of proteoglycan and attenuated cartilage destruction in rabbit arthritic knees [14]. In the present study, we found that resveratrol was able to increase Alcian Blue staining intensity and biochemical content (GAG and HYP), and up-regulate expression of NP matrix anabolism-related molecules (SOX-9, aggrecan, and collagen II) at both gene and protein levels in a dose-dependent manner, indicating that resveratrol has similar protective effects on disc NP matrix biosynthesis under the mechanical overloading.

Previous studies have showed that resveratrol plays its beneficial role in aging, inflammation, and matrix metabolism through activation of the lysine deacetylase, sirtuin 1 (SIRT1), the cAMP pathway, or AMP-activated protein kinase [31]. In the present study, we found that though the activity of the PI3K/Akt pathway in the mechanical compression group is obviously lower than in the control group, addition of the resveratrol significantly increased the activity of the PI3K/Akt pathway in a dose-dependent manner under the mechanical compression. In light of the corresponding alteration of NP matrix biosynthesis after the addition of the resveratrol under the mechanical overloading, we deduce that resveratrol may enhance NP matrix synthesis through activating the PI3K/Akt pathway under this high-magnitude compression.

Among previous disc studies, several animal species have been used to investigate disc degeneration such as rat, mouse, rabbit, bovine, porcine, and dog [32]. The present study used the discs from the immature pig. Although the pig is suitable to study human disc degeneration due to its similar disc changes in the aging process [33], Alini et al. [34] reported that cow and sheep are more similar to human than porcine in terms of disc development, and that study also emphasized that the existence of notochordal cells in certain animal’s disc (i.e. rodent animal species and pig) may limit the translation of experimental results to adult human situation. Hence, the results presented in the present study should be interpreted carefully when translated to disc biology of adults. Additionally, because we mainly aimed to investigate NP matrix under mechanical load, the adjacent AF and CEP were not investigated here, which is also a limitation of the present study because these three parts are structurally connected *in vivo*.

In conclusion, the present study confirms again that mechanical overloading can suppress disc NP matrix biosynthesis. Meanwhile, the present study demonstrates that resveratrol can enhance NP matrix biosynthesis under mechanical overloading through activating the PI3K/Akt pathway. The present study directly provides that resveratrol may be a promising drug for regenerating mechanical overloading-induced disc degeneration.

## Abbreviations

ADAMTS-4: A Disintegrin And Metalloprotease Thrombospondin Motify-4
AF: annulus fibrosus
CEP: cartilage endplate
DMMB: dimethylmethylene blue
DMEM: Delbecco’s Modified Eagle’s Medium
GAPDH: Glyceraldehyde-3 Phosphate Dehydrogenase
GAG: glycosaminoglycan
HYP: hydroxyproline
IDD: intervertebral disc degeneration
IVD: intervertebral disc
LSD: Lactic Dehydrogenase
MMP-3: Matrix Metallo Preteinases-3
MMP-13: Matrix Metallo Preteinases-13
NP: nucleus pulposus
SOX-9: SRY-related High Mobility Group-box Gene 9

## References

[1] BorensteinD. (1991) Low back pain: epidemiology, etiology, diagnostic evaluation, and therapy. Curr. Opin. Rheumatol. 3, 207–2171829622

[2] ManchikantiL., SinghV., FalcoF.J., BenyaminR.M. and HirschJ.A. (2014) Epidemiology of low back pain in adults. Neuromodulation: J. Int. Neuromodulation Soc. 17, 3–1010.1111/ner.1201825395111

[3] VassilakiM. and HurwitzE.L. (2014) Insights in public health: perspectives on pain in the low back and neck: global burden, epidemiology, and management. Hawai’i J. Med. Public Health: a J. Asia Pacific Med. Public Health 73, 122–126PMC399823224765562

[4] LeeC.R., IatridisJ.C., PovedaL. and AliniM. (2006) In vitro organ culture of the bovine intervertebral disc: effects of vertebral endplate and potential for mechanobiology studies. Spine 31, 515–5221650854410.1097/01.brs.0000201302.59050.72PMC7187957

[5] RobertsS. (2002) Disc morphology in health and disease. Biochem. Soc. Trans. 30, 864–8691244093410.1042/bst0300864

[6] CabrajaM., EndresM., AbbushiA., ZenclussenM., BlechschmidtC., LemkeA.J. (2013) Effect of degeneration on gene expression of chondrogenic and inflammatory marker genes of intervertebral disc cells: a preliminary study. J. Neurosurg. Sci. 57, 307–31624091434

[7] PockertA.J., RichardsonS.M., Le Maitre CLLyon M, DeakinJ.A., ButtleD.J. (2009) Modified expression of the ADAMTS enzymes and tissue inhibitor of metalloproteinases 3 during human intervertebral disc degeneration. Arthritis Rheum. 60, 482–4911918049310.1002/art.24291

[8] SettonL.A. and ChenJ. (2006) Mechanobiology of the intervertebral disc and relevance to disc degeneration. J. Bone Jt. Surg. 88, 52–5710.2106/JBJS.F.0000116595444

[9] HsiehA.H. and TwomeyJ.D. (2010) Cellular mechanobiology of the intervertebral disc: new directions and approaches. J. Biomech. 43, 137–1451982815010.1016/j.jbiomech.2009.09.019PMC2813313

[10] ChanS.C., FergusonS.J. and Gantenbein-RitterB. (2011) The effects of dynamic loading on the intervertebral disc. Eur. Spine J. 20, 1796–18122154166710.1007/s00586-011-1827-1PMC3207351

[11] LiP., GanY., WangH., ZhangC., WangL., XuY. (2016) Dynamic compression effects on immature nucleus pulposus: a study using a novel intelligent and mechanically active bioreactor. Int. J. Med. Sci. 13, 225–2342694158310.7150/ijms.13747PMC4773287

[12] CottartC.H., Nivet-AntoineV. and BeaudeuxJ.L. (2014) Review of recent data on the metabolism, biological effects, and toxicity of resveratrol in humans. Mol. Nutr. Food Res. 58, 7–212374085510.1002/mnfr.201200589

[13] YangS.D., MaL., YangD.L. and DingW.Y. (2016) Combined effect of 17beta-estradiol and resveratrol against apoptosis induced by interleukin-1beta in rat nucleus pulposus cells via PI3K/Akt/caspase-3 pathway. Peer J. 4, e16402682400010.7717/peerj.1640PMC4730868

[14] LiX., PhillipsF.M., AnH.S., EllmanM., ThonarE.J., WuW. (2008) The action of resveratrol, a phytoestrogen found in grapes, on the intervertebral disc. Spine 33, 2586–25951901154010.1097/BRS.0b013e3181883883PMC2905225

[15] LiM., GuQ., ChenM., ZhangC., ChenS. and ZhaoJ. (2017) Controlled delivery of icariin on small intestine submucosa for bone tissue engineering. Mater. Sci. Eng. C Mater. Biol. Appl. 71, 260–2672798770710.1016/j.msec.2016.10.016

[16] LiS.T., LiuY., ZhouQ., LueR.F., SongL., DongS.W. (2014) A novel axial-stress bioreactor system combined with a substance exchanger for tissue engineering of 3D constructs. Tissue Eng. Part C, Methods 20, 205–2142382209210.1089/ten.TEC.2013.0173

[17] HaschtmannD., StoyanovJ.V., EttingerL., NolteL.P. and FergusonS.J. (2006) Establishment of a novel intervertebral disc/endplate culture model: analysis of an ex vivo in vitro whole-organ rabbit culture system. Spine (Phila Pa 1976) 31, 2918–29251713922210.1097/01.brs.0000247954.69438.ae

[18] FarndaleR.W., SayersC.A. and BarrettA.J. (1982) A direct spectrophotometric microassay for sulfated glycosaminoglycans in cartilage cultures. Connect. Tissue Res. 9, 247–248621520710.3109/03008208209160269

[19] RasweilerJ.J.t., CretekosC.J. and BehringerR.R. (2009) Alcian blue/alizarin red staining of cartilage and bone of short-tailed fruit bat (Carollia perspicillata). Cold Spring Harb. Protoc. 2009. 3 10.1101/pdb.prot5166 pdb prot5166.20147101

[20] LiP., GanY., XuY., LiS., SongL., LiH. (2016) Osmolarity affects matrix synthesis in the nucleus pulposus associated with the involvement of MAPK pathways: A study of ex vivo disc organ culture system. J. Orthop. Res. 34, 1092–11002657604310.1002/jor.23106

[21] GruberH.E. and HanleyE.N.Jr (2003) Recent advances in disc cell biology. Spine (Phila Pa 1976) 28, 186–1931254493810.1097/00007632-200301150-00017

[22] LotzJ.C. and KimA.J. (2005) Disc regeneration: why, when, and how. Neurosurg. Clin. N. Am. 16, 657–663, vii1632628910.1016/j.nec.2005.06.004

[23] JungerS., Gantenbein-RitterB., LezuoP., AliniM., FergusonS.J. and ItoK. (2009) Effect of limited nutrition on in situ intervertebral disc cells under simulated-physiological loading. Spine (Phila Pa 1976) 34, 1264–12711945500110.1097/BRS.0b013e3181a0193d

[24] GantenbeinB., Illien-JungerS., ChanS.C., WalserJ., HaglundL., FergusonS.J. (2015) Organ culture bioreactors–platforms to study human intervertebral disc degeneration and regenerative therapy. Current Stem Cell Res. Ther. 10, 339–35210.2174/1574888x10666150312102948PMC443786125764196

[25] ZhangF., ZhaoX., ShenH. and ZhangC. (2016) Molecular mechanisms of cell death in intervertebral disc degeneration (Review). Int. J. Mol. Med. 37, 1439–14482712148210.3892/ijmm.2016.2573PMC4866972

[26] WangF., CaiF., ShiR., WangX.H. and WuX.T. (2016) Aging and age related stresses: a senescence mechanism of intervertebral disc degeneration. Osteoarthritis Cartilage 24, 398–4082645595810.1016/j.joca.2015.09.019

[27] MaK.G., ShaoZ.W., YangS.H., WangJ., WangB.C., XiongL.M. (2013) Autophagy is activated in compression-induced cell degeneration and is mediated by reactive oxygen species in nucleus pulposus cells exposed to compression. Osteoarthritis Cartilage 21, 2030–20382412049010.1016/j.joca.2013.10.002

[28] WalterB.A., KoreckiC.L., PurmessurD., RoughleyP.J., MichalekA.J. and IatridisJ.C. (2011) Complex loading affects intervertebral disc mechanics and biology. Osteoarthritis Cartilage 19, 1011–10182154984710.1016/j.joca.2011.04.005PMC3138834

[29] ElmaliN., EsenkayaI., HarmaA., ErtemK., TurkozY. and MizrakB. (2005) Effect of resveratrol in experimental osteoarthritis in rabbits. Inflammation Res.: Official J. Eur. Histamine Res. Soc. 54, 158–16210.1007/s00011-004-1341-615883738

[30] ElmaliN., BaysalO., HarmaA., EsenkayaI. and MizrakB. (2007) Effects of resveratrol in inflammatory arthritis. Inflammation 30, 1–61711511610.1007/s10753-006-9012-0

[31] NwachukwuJ.C., SrinivasanS., BrunoN.E., ParentA.A., HughesT.S., PollockJ.A. (2014) Resveratrol modulates the inflammatory response via an estrogen receptor-signal integration network. eLife 3, e020572477176810.7554/eLife.02057PMC4017646

[32] LotzJ.C. (2004) Animal models of intervertebral disc degeneration: lessons learned. Spine (Phila Pa 1976) 29, 2742–27501556492310.1097/01.brs.0000146498.04628.f9

[33] ChoH., ParkS.H., LeeS., KangM., HastyK.A. and KimS.J. (2011) Snapshot of degenerative aging of porcine intervertebral disc: a model to unravel the molecular mechanisms. Exp. Mol. Med. 43, 334–3402149901210.3858/emm.2011.43.6.036PMC3128911

[34] AliniM., EisensteinS.M., ItoK., LittleC., KettlerA.A., MasudaK. (2008) Are animal models useful for studying human disc disorders/degeneration? Eur. Spine J. 17, 2–191763273810.1007/s00586-007-0414-yPMC2365516

